# The world’s first glyphosate-resistant case of *Avena fatua* L. and *Avena sterilis* ssp. *ludoviciana* (Durieu) Gillet & Magne and alternative herbicide options for their control

**DOI:** 10.1371/journal.pone.0262494

**Published:** 2022-01-12

**Authors:** Bhagirath Singh Chauhan

**Affiliations:** 1 The Centre for Crop Science, Queensland Alliance for Agriculture and Food Innovation (QAAFI) and School of Agriculture and Food Sciences (SAFS), The University of Queensland, Gatton, QLD, Australia; 2 Department of Agronomy, Chaudhary Charan Singh Haryana Agricultural University, Hisar, Haryana, India; Anhui Agricultural University, CHINA

## Abstract

*Avena fatua* and *A*. *ludoviciana* (commonly known as wild oats) are the most problematic winter grass species in fallows and winter crops in the northeast region of Australia. A series of experiments were conducted to evaluate the performance of glyphosate and alternative post-emergence herbicides on *A*. *fatua* and *A*. *ludoviciana*. This study reports the world’s first glyphosate-resistant (GR) biotypes of *A*. *fatua* and *A*. *ludoviciana*. The glyphosate dose required to kill 50% of the plants (LD_50_) and to reduce 50% of the biomass (GR_50_) for the GR biotype of *A*. *fatua* was 556 g a.e./ha and 351 g a.e./ha, respectively. These values for *A*. *ludoviciana* were 848 g a.e./ha and 289 g a.e./ha. Regardless of the growth stage (3–4 or 6–7 leaf stages), clethodim (120 g a.i./ha), haloxyfop (78 g a.i./ha), pinoxaden (20 g a.i./ha), and propaquizafop (30 g a.i./ha) were the best alternative herbicide options for the control of *A*. *fatua* and *A*. *ludoviciana*. The efficacy of butroxydim (45 g a.i./ha), clodinafop (120 g a.i./ha), imazamox + imazapyr (36 g a.i./ha), and paraquat (600 g a.i./ha) reduced at the advanced growth stage. Glufosinate (750 g a.i./ha), flamprop (225 g a.i./ha), and pyroxsulam + halauxifen (20 g a.i./ha) did not provide effective control of *Avena* species. This study identified alternative herbicide options to manage GR biotypes of *A*. *fatua* and *A*. *ludoviciana*.

## Introduction

Weeds are an important biological constraint to the production of grains crops in Australia. They cost Australian grain growers more than AUD 3.3 billion [1]. *Avena fatua* L. and *A*. *sterilis* ssp. *ludoviciana* (Durieu) Gillet & Magne (hereafter, *A*. *ludoviciana*) (both known as wild oats in Australia) are the second most important grass weed in Australia, causing a revenue loss of more than AUD 28 million per annum to grain growers [1]. In the northeast grain region of Australia, *Avena* species are the top-ranked weed in terms of infested area (630,000 ha). A recent study reported that 15 to 16 plants/m^2^ of *A*. *fatua* and *A*. *ludoviciana* were enough to cause a 50% yield loss in wheat [2].

*Avena fatua* is most common in Southern Australia and *A*. *ludoviciana* is dominant in eastern Australia [3]. However, mixed populations of both species exist in the northeast region of Australia. Both species are difficult to differentiate at the vegetative phase because of very similar morphological characters. However, they can be distinguished at maturity as seeds of *A*. *ludoviciana* shatter in pairs and *A*. *fatua* seeds shatter singularly [4]. In the same study, *A*. *fatua* produced a greater number of seeds (480 seeds/plant) than *A*. *ludoviciana* (420 seeds/plant) and both species were able to produce a considerable number of seeds at 60% of the water holding capacity. However, seeds do not persist long on the soil surface. For example, 50% of the seeds of *A*. *fatua* and *A*. *ludoviciana* were found to be decayed in 6 months [5]. Another study reported that although May-emerged cohorts of *A*. *ludoviciana* produced a higher number of seeds than June- and July-emerged cohorts, late cohorts produced sufficient seeds for reinfestation [6].

A fallow phase in winter or summer is very common in northeastern Australia, depending on soil moisture [7, 8]. Without crop competition, fallow fields are prone to weed infestation. Growers rely on non-selective herbicides (e.g., glyphosate) to control weeds during the fallow phase. However, the continuous use of glyphosate has led to the evolution of glyphosate-resistant (GR) weeds [9]. The world’s first case of GR *A*. *fatua* and *A*. *ludoviciana* was registered in 2018 from the northeastern region of Australia [9]. However, details are not available in the literature on the dose-response of those biotypes to glyphosate.

Alternative herbicide programs need to be developed to manage GR biotypes of *Avena* species. Therefore, there is a need to evaluate the performance of different post-emergence herbicides for the control of GR *Avena* species. As shown in several studies [10, 11], herbicide efficacy can be affected by the growth stage of the weed. Therefore, there is a need to evaluate the performance of post-emergence herbicides at different growth stages of *Avena* species.

Knowledge of effective post-emergent herbicides can be used to develop effective management programs for GR *Avena* species in fallows. Therefore, a series of pot experiments were conducted to evaluate the response of *A*. *fatua* and *A*. *ludoviciana* to glyphosate and alternative post-emergence herbicides. The aims of this study were (i) to confirm glyphosate resistance in *A*. *fatua* and *A*. *ludoviciana*, and (ii) to evaluate the response of both species to alternative post-emergent herbicides.

## Material and methods

### Seed collection

Seeds of one biotype each of *A*. *fatua* and *A*. *ludoviciana* were collected in October 2017 from a chickpea (*Cicer arietinum* L.) field (Warialda, New South Wales; 29.6075°S, 150.6888°E) infested with both species. In winter 2018 (May to November), seeds of both species were planted separately in pots in the same environment at the Gatton research farm of the University of Queensland, Queensland, Australia. Plants were regularly watered and the seeds that were collected from these plants were used for subsequent experiments. These biotypes were named the GR biotypes of *A*. *fatua* and *A*. *ludoviciana*. These biotypes were not suspected of resistance to glyphosate. Seeds of a glyphosate-susceptible (GS) biotype of *A*. *ludoviciana* were collected in October 2017 from a wheat (*Triticum aestivum* L.) field in St. George, Queensland (28.0343°S, 148.5740°E). The straight line distance between the two locations (Warialda and St George) is about 250 km. Seeds of a GS biotype of *A*. *fatua* were collected from a chickpea field in November 2017 from Moree, New South Wales (29.4455°S, 149.8577°E). The straight line distance between the two locations (Warialda and Moree) is about 70 km. Permission to collect seeds of both biotypes was taken from the landlord. The names (GR and GS) were given after confirming their resistance status (see the next section). The biotype was considered resistant when at least 20% of seedlings survived the field recommended rate of glyphosate.

### Response to glyphosate dose

In the experiment, two biotypes (GR and GS) of each species were used. Pot experiments were conducted three times in 2019 (June to October) to evaluate the response of *A*. *fatua* and *A*. *ludoviciana* biotypes to different doses of glyphosate. Twelve seeds of each biotype were planted in 20-cm diameter pots filled with a commercial potting mix (Centenary landscape, Mt Ommaney, Queensland). Immediately after emergence, plants were thinned to keep 8 plants/pot.

Glyphosate at different doses (185, 370, 740, 1480, 2960, and 5920 g a.e./ha) was sprayed at the 3–4 leaf stage of each biotype. The maximum recommended dose of glyphosate for *Avena* species control in Australia is 540 g a.e./ha Herbicide was applied using a research track sprayer, which delivered 108 L/ha spray solution through flat ban nozzles (TeeJet XR 110015). There was also a nontreated control treatment for each biotype. Pots were regularly watered using an automated sprinkler system; however, plants were not watered for 24 h after herbicide treatment.

In each experimental run, there were three replications of each treatment and the experiment was conducted using a randomized complete block design. Seedling survival data was taken 28 days after herbicide treatment with the criterion of at least one new leaf on the plants. Survived plants were cut at the base, placed in paper bags, and oven-dried at 70°C for 72 h. Samples were weighed and presented as the biomass of the nontreated control.

### Response to growth stage and post-emergence herbicides

Seeds (12) of the GR biotype of *A*. *fatua* and *A*. *ludoviciana* were planted in 20-cm diameter pots. Plants were thinned to 8 plants/pot immediately after emergence. A range of post-emergence herbicides at recommended doses (Table 1) was sprayed at the 3–4 leaf (small stage) and 6–7 leaf stage (large stage) of each species. There was a nontreated control for each leaf stage and species. Survival and biomass data were determined at 28 days after spray as mentioned previously. This experiment was conducted in a randomized complete block design with three replications of each experiment. The experiment was conducted during the winter season of 2019 and repeated during the winter season of 2020.

**Table 1:** Post-emergence herbicides, their recommended doses, and adjuvants used to spray *Avena fatua* and *A*. *ludoviciana* at two growth stages (small plants: 3–4 leaf stage; large plants: 6–7 leaf stage).

Treatments	Herbicide MOA	Dose (g ai/ha)	Adjuvants
Control	-	-	-
Butroxydim	Inhibition of acetyl CoA carboxylase (ACCase)	45	1% Supercharge
Clethodim	Inhibition of ACCase	120	1% Supercharge
Clodinafop	Inhibition of ACCase	20	0.5% Hasten
Flamprop	Unknown	225	-
Glufosinate	Inhibition of glutamine synthetase	750	-
Haloxyfop	Inhibition of ACCase	78	1% Hasten
Imazamox + imazapyr	Inhibition of acetolactase synthase (ALS)	36	1% Hasten
Paraquat	Inhibitors of photosystem-I	600	1% BS1000
Pinoxaden	Inhibition of ACCase	20	0.5% Adigor
Propaquizafop	Inhibition of ACCase	30	0.5% Hasten
Pyroxsulam + halauxifen	Inhibition of ALS + disrupters of plant cell growth	20	0.5% BS1000

### Response to imazamox + imazapyr dose

There is anecdotal evidence that the commercial mixture of imazamox (3.3% a.i.) and imazapyr (1.5% a.i.) provides differential control of *A*. *fatua* and *A*. *ludoviciana*. Therefore, a pot trial was conducted to evaluate the response of *A*. *fatua* and *A*. *ludoviciana* to different doses (0, 9, 18, 36, 72, and 144 g a.i./ha) of this commercial herbicide. Seeds were planted as described above and plants were sprayed at the 4–5 leaf stage. The experiment was conducted in a randomized complete block design with three replications of each treatment. Survival and biomass data were taken 28 days after herbicide treatment as described above.

### Statistical analysis

Experimental runs were combined as there was no treatment by experimental run interaction [12]. In the dose-response experiments (3.2 and 3.4), the herbicide doses required to kill 50% of the plants (LD_50_) and to reduce 50% of the biomass (GR_50_) were calculated by fitting a three-parameter log-logistic model to the survival and biomass data, respectively (SigmaPlot 14.0). The model was

$$S=a/\left[1+{\left(d/H_{50}\right)}^{b}\right]$$

In this model, *S* is the survival or biomass value at herbicide dose ‘*d*’, *a* is the maximum seedling survival or biomass, *H*_*50*_ is the herbicide dose (g a.i. or a.e./ha) required for 50% reduction in plant survival (LD_50_) or biomass (GR_50_), and *b* is the slope of the model. Resistance index (RI) was calculated as the ratio between the LD_50_ or GR_50_ of each resistant biotype and the LD_50_ or GR_50_ of the susceptible biotype. For the post-emergence and growth stage experiment, survival and biomass data were analyzed separately for each leaf stage using one-way analysis of variance (ANOVA). Means were compared using the least significant difference (LSD) at 0.05 probability.

## Results and discussion

### Response to glyphosate dose

The dose-response study confirmed resistance in the suspected biotype of *A*. *fatua* and *A*. *ludoviciana* (Fig 1). No seedlings of the glyphosate-susceptible (GS) biotype of *A*. *fatua* survived glyphosate at 740 g a.e./ha; however, greater than 26% of seedlings of the GR biotype survived at this rate (Fig 1A). Although the maximum recommended dose of glyphosate for *Avena* species control in Australia is 540 g a.e./ha, the recommendation for control of some other weeds in fallows is 740 g a.e./ha. Growers rarely use the lower glyphosate dose recommended for *Avena* species. The LD_50_ for the GS biotype of *A*. *fatua* was 384 g a.e./ha, whereas the LD_50_ for the GR biotype was 556 g a.e./ha (Table 2). The GR50 for the GS biotype of *A*. *fatua* was 288 g a.e./ha, whereas this value for the GR biotype was 351 g a.e./ha (Fig 1B and Table 2). Although the LD_50_ and GR_50_ values of the GR biotype were only 1.2 to 1.5-fold greater than the GS biotype, the results confirmed evolution of glyphosate resistance has occurred in *A*. *fatua*. This is the first global case of GR *A*. *fatua* (Heap 2021).

**Fig 1:** Effect of glyphosate dose on survival (%) (a and b) and biomass (percent of nontreated control) (c and d) of glyphosate-resistant (GR) and glyphosate-susceptible (GS) biotypes of *Avena fatua* (a and c) and *A*. *ludoviciana* (b and d). Plants were sprayed at the 3–4 leaf stage of each biotype.

**Table 2:** Estimated glyphosate dose required to kill 50% of the plants (LD_50_) of *Avena fatua* and *A*. *ludoviciana*, glyphosate dose required to reduce their biomass by 50% (GR_50_), and resistance indices (RI).

Species	Biotype	LD_50_	RI	GR_50_	RI
		(g a.e./ha)		(g a.e./ha)	
*Avena fatua*	Glyphosate-resistant	556	1.45	351	1.22
*A*. *fatua*	Glyphosate-susceptible	384		288	
*Avena ludoviciana*	Glyphosate-resistant	848	3.25	289	1.55
*A*. *ludoviciana*	Glyphosate-susceptible	261		187	

RI were calculated as the ratio between the LD_50_ or GR_50_ of each resistant population and the LD_50_ or GR_50_ of the susceptible control.

No seedlings of the GS biotype of *A*. *ludoviciana* survived glyphosate at 370 g a.e./ha; however, 73% of seedlings of the GR biotype of *A*. *ludoviciana* survived this herbicide rate (Fig 1C). At the commonly used glyphosate dose (740 g a.e./ha), 79% of seedlings of the GR biotype survived. The LD_50_ for the GS biotype of *A*. *ludoviciana* was 261 g a.e./ha, whereas the LD_50_ for the GR biotype was 848 g a.e./ha (Table 2), which was 3.3 times greater than the GS biotype. The GR_50_ for the GS biotype of *A*. *ludoviciana* was 187 g a.e./ha, whereas this value for the GR biotype was 289 g a.e./ha (Fig 1D and Table 2). This study also reported the first global case of GR *A*. *ludoviciana* [9].

Studies have reported glyphosate resistance in several weed species throughout Australia and other parts of the world [13–15]. In previous studies, very high levels of resistance were reported in GR biotypes compared with GS biotypes; for example, 8- to 13-fold glyphosate resistance was reported in a biotype of *Conyza canadensis* [14]. In the current study, however, only 1.5 to 3.3-fold glyphosate resistance was found in the GR biotype of *A*. *fatua* and *A*. *ludoviciana*. This low level of resistance to glyphosate suggests that both *Avena* species have initiated evolving resistance to glyphosate, and this level of resistance could increase dramatically in the next few years. Therefore, there is a need to screen several populations of both species of *Avena* from the northeast region of Australia to glyphosate.

### Response to growth stage and post-emergence herbicides

In general, both weed species responded similarly to different post-emergence herbicides. Clethodim, haloxyfop, pinoxaden, and propaquizafop were the best alternative herbicide options for the control of *A*. *fatua* and *A*. *ludoviciana*. Regardless of the growth stage, these herbicides provided complete control of both *Avena* species (Table 3). Butroxydim provided complete control of *A*. *fatua* and *A*. *ludoviciana* when sprayed at the 3–4 leaf stage. Delaying its spray till the 6–7 leaf stage resulted in 38 and 7% survival of *A*. *fatua* and *A*. *ludoviciana* seedlings, respectively. These seedlings, however, produced only 15% and 2% biomass of their respective nontreated control, respectively. The next best herbicides were clodinafop and paraquat, which resulted in 4 to 5% and 5 to 8% survival of *Avena* species, respectively, when sprayed at the 3–4 leaf stage. Delaying their application to the 6–7 leaf stage resulted in a greater number of survivors. Regardless of the growth stage, compared with *A*. *fatua*, a greater number of *A*. *ludoviciana* seedlings survived the application of imazamox + imazapyr (Table 3). However, their seedlings produced only 1 to 3% biomass of their nontreated control treatments. Flamprop and pyroxsulam + halauxifen did not provide any control of *A*. *fatua* and *A*. *ludoviciana*. Although glufosinate reduced biomass by 72 to 83% compared to nontreated control treatments, 48 to 83% of seedlings of *A*. *fatua* and *A*. *ludoviciana* survived the application of glufosinate.

**Table 3:** Performance of different post-emergence herbicides on seedling survival (%) and biomass (g/pot) of *Avena fatua* and *A*. *ludoviciana* when sprayed at two growth stages (small plants: 3–4 leaf stage; large plants: 6–7 leaf stage).

Treatments	*Avena fatua*				*Avena ludoviciana*			
	Small plants (3–4 leaves)		Large plants (6–7 leaves)		Small plants (3–4 leaves)		Large plants (6–7 leaves)	
	Survival (%)	Biomass (g/pot)	Survival (%)	Biomass (g/pot)	Survival (%)	Biomass (g/pot)	Survival (%)	Biomass (g/pot)
Control	100.0	5.55	100.0	6.39	100.0	7.12	100.0	8.53
Butroxydim	0	0 (100)	38.1	1.01 (84)	0	0 (100)	6.7	0.21 (98)
Clethodim	0	0 (100)	0	0 (100)	0	0 (100)	0	0 (100)
Clodinafop	3.7	0.08 (99)	21.3	0.40 (94)	5.0	0.14 (98)	16.7	0.54 (94)
Flamprop	95.5	3.84 (31)	100.0	5.17 (19)	100.0	6.18 (13)	100.0	7.59 (11)
Glufosinate	48.3	1.27 (77)	80.0	1.79 (72)	50.0	1.20 (83)	73.6	1.73 (80)
Haloxyfop	0	0 (100)	0	0 (100)	0	0 (100)	0	0 (100)
Imazamox + imazapyr	10.0	0.05 (99)	15.2	0.10 (98)	23.3	0.22 (97)	33.3	0.29 (97)
Paraquat	8.3	0.14 (94)	16.9	0.39 (94)	5.0	0.06 (99)	7.2	0.11 (99)
Pinoxaden	0	0 (100)	0	0 (100)	0	0 (100)	0	0 (100)
Propaquizafop	0	0 (100)	0	0 (100)	0	0 (100)	0	0 (100)
Pyroxsulam + halauxifen	100.0	2.26 (59)	100.0	3.26 (49)	81.7	2.14 (70)	100.0	2.60 (70)
LSD_0.05_	17.4	1.10	26.9	1.45	21.2	1.49	15.9	1.821

Values in parentheses are percent reductions of their respective nontreated control treatment.

Acetyl-CoA carboxylase (ACCase)-inhibiting (Group 1) herbicides have been widely used to selectively control *Avena* species in a range of crops across several continents. In the present study, all herbicides, except clodinafop, from this group provided excellent control of both *Avena* species. Continued and widespread use of ACCase-inhibiting herbicides has resulted in the evolution of resistance in *Avena* species in different countries [16–18]. A survey in Western Australian cropping fields revealed that almost 50% of *Avena* species populations displayed resistance to the commonly used ACCase-inhibiting herbicides [18]. These results suggest that ACCase-inhibiting herbicides need to be rotated with herbicides with different modes of action to delay the evolution of resistance in weeds. The present study identified effective ACCase-inhibiting herbicides from subgroups ‘dim’ (butroxydim and clethodim), ‘fop’ (haloxyfop and propaquizafop), and ‘den’ (pinoxaden). Rotating herbicides from different subgroups can play a key role in managing GR *Avena* species.

Although 10 to 33% of *A*. *fatua* and *A*. *ludoviciana* plants survived the application of the commercial mixture of imazamox + imazapyr [acetolactase synthase (ALS)-inhibiting herbicides], these plants produced only 1 to 3% biomass of the control plants. In this study, the biomass was measured 28 days after spray. In the field, surviving plants may continue to grow and produce seeds. Therefore, the application of this herbicide should be followed by a sequential treatment of another herbicide or a non-chemical tool. No survey has been conducted in northeast Australia to screen *Avena* species against this herbicide mixture, but a survey conducted in Western Australia reported only one population of *Avena* species was resistant to imazamox + imazapyr [18]. The previous study, however, used only half the rate (18 g a.i./ha) than what used in the current study (36 g a.i./ha).

Paraquat, inhibitors of photosystem-I, was also found to be effective in controlling both species of *Avena*. Less than 20% of seedlings survived the application of paraquat, which produced only 1 to 6% biomass of the nontreated plants (Table 3). Australian growers visually recognize resistance in the field at about 20% survival and may consider alternative management options [18]. The survey conducted in Western Australia reported that all populations (98) of *Avena* species were susceptible to paraquat at 250 g a.i./ha [18]. In the current study, paraquat was used at 600 g a.i./ha, suggesting that the performance of paraquat needs to be evaluated on several populations of *Avena* species from the northeast region of Australia.

Glufosinate, an inhibitor of glutamine synthetase, is a nonselective post-emergence herbicide with a broad spectrum of activity [19]. It is recommended for the control of *Avena* species; however, the present study experienced poor efficacy of glufosinate, resulting in 48 to 80% survival of *A*. *fatua* and *A*. *ludoviciana* plants (Table 3). Poor control of *Avena* species can occur when relative humidity is low at the time of glufosinate spray. For example, exposure to >95% relative humidity, as opposed to 40% relative humidity, increased glufosinate efficacy on *A*. *fatua* in Western Canada, suggesting that poor control of *A*. *fatua* with glufosinate could be due to application during conditions of low relative humidity [19]. In the present study, relative humidity was not measured but a nearby weather station showed >60% relative humidity during June, July, and August of 2019 and 2020 (bom.gov.au). Temperature can also affect glufosinate efficacy [20], however, the effect of temperature on glufosinate efficacy was not evaluated in the current study.

Flamprop and the commercial mixture of pyroxsulam + halauxifen did not provide any control of either species of *Avena* (Table 3). These results suggest the possibility of evolution of resistance to these herbicides in these biotypes of *Avena* species. Therefore, future studies should screen populations of *Avena* species from northeast Australia to flamprop and pyroxsulam + halauxifen. In a survey, resistance to flamprop was detected for the first time in Western Australia, in which eight populations (out of 104) of *Avena* species survived flamprop at 270 g a.i./ha [18].

### Response to imazamox + imazapyr dose

In the previous experiment, compared with *A*. *fatua*, a greater number of *A*. *ludoviciana* seedlings survived imazamox + imazapyr at 36 g a.i./ha (Table 3). This experiment evaluated the response of *A*. *fatua* and *A*. *ludoviciana* to different doses of the commercial mixture. The LD_50_ values for both species were similar (36.4 to 37.1 g a.i./ha) (Fig 2A). The difference in survival was observed only at the recommended rate (36 g a.i./ha). GR_50_ values, however, were different between the two species. The GR_50_ value for *A*. *ludoviciana* was 29.8 g a.i./ha, whereas this value for *A*. *fatua* was only 20.6 g a.i./ha (Fig 2B). These results could mean that the *A*. *ludoviciana* biotype was more tolerant to imazamox + imazapyr than the *A*. *fatua* biotype. These results could also be seen as supporting anecdotal evidence that this herbicide mixture provides more effective control of *A*. *fatua* than *A*. *ludoviciana*. This hypothesis needs to be confirmed using several populations of both species. Such responses may result in the shift towards *A*. *ludoviciana* populations in a mixed-infested field.

**Fig 2:** Effect of imazamox and imazapyr (a commercial mixture) dose on survival (%) (a) and biomass (percent of nontreated control) (b) of the glyphosate-resistant biotypes of *Avena fatua* (Afat) and *A*. *ludoviciana* (Alud). Plants were sprayed at the 4–5 leaf stage of each species.

## Conclusions

This study reported the world’s first glyphosate-resistant cases of *A*. *fatua* and *A*. *ludoviciana*. Winter fallows are common in the northeast region of Australia, in which growers rely on glyphosate for weed control. Therefore, there is a need to screen populations of both species of *Avena* to glyphosate. There is a possibility of the occurrence of more cases of GR *Avena* species. Future research should evaluate the mechanism of resistance (target-site or non-target site) in *Avena* species. This research identified alternative herbicide options to manage GR *Avena* species. ACCase-inhibiting herbicides were particularly effective against *Avena* species and if used judiciously, these herbicides could play an important role in managing GR populations of *Avena* species. Glufosinate did not provide effective control of either species of *Avena*. Therefore, there is a need to compare these biotypes with other biotypes of *Avena* species to understand the reason for the poor glufosinate efficacy. Future research should also evaluate differential responses of *A*. *fatua* and *A*. *ludoviciana* populations to different herbicides, especially to imazamox + imazapyr.
